The article "Clinical Efficacy of Creatine Phosphate Sodium and/or Vitamin C in the Treatment of Children with Viral Myocarditis: A Meta-Analysis" was retracted in 2023. Reasons: suspected computer-generated content; unreliable results or conclusions; concerns about the data; concerns about the results or conclusions.

# Clinical Efficacy of Creatine Phosphate Sodium and/or Vitamin C in the Treatment of Children with Viral Myocarditis: A Meta-Analysis

**DOI:** 10.1155/2022/3840891

**Published:** 2022-08-10

**Authors:** Qiyu Li, Siyuan Liu, Xuemei Ma, Jiaping Yu

**Affiliations:** Department of Pediatrics, General Hospital of Northern Theater Command, No. 5 Guangrong Street, Heping District, Shenyang 110812, China

## Abstract

**Background:**

This study performed a meta-analysis to explore the clinical efficacy of creatine phosphate sodium (CPS) and/or vitamin C for viral myocarditis (VMC) in children, to provide guidance for its clinical treatment.

**Methods:**

A literature search was performed on PubMed, Web of Science, Embase, China National Knowledge Infrastructure, and Wanfang databases to obtain published clinical randomized controlled trials (RCTs) on CPS and/or vitamin C for VMC in children, with a time span from 2013 to 2022. Relevant data was extracted and meta-analysis was performed using the statistical software Stata 16.0.

**Results:**

A total of 723 studies were retrieved and 19 studies were finally included for meta-analysis, with a total of 1,957 patients. The meta-analysis results showed that the observation group (conventional treatment + CPS and/or vitamin C) was superior to the control group (conventional treatment alone) in treatment effective rate (OR = 3.60, 95% CI (2.55, 5.07), and *P* < 0.001). Additionally, the observation group had lower levels of cardiac troponin-I (SMD = − 2.63, 95% CI (− 3.51, − 1.76), and *P* < 0.001), creatine kinase isoenzyme (SMD = −2.78, 95% CI (− 3.53, − 2.03), and *P* < 0.001), lactate dehydrogenase (SMD = −1.95, 95% CI (− 2.49, − 1.42), and *P* < 0.001), aspartate aminotransferase (SMD = −0.87, 95% CI (− 1.84, 0.09), and *P* = 0.076), tumor necrosis factor-*α* (SMD = −3.90, 95% CI (− 4.47, − 3.06), and *P* < 0.001), and higher superoxide dismutase levels (SMD = 2.48, 95% CI (1.64, 3.33), and *P* < 0.001). Except aspartate aminotransferase, there were significant differences between the two groups in the other parameters.

**Conclusion:**

CPS and/or vitamin C treatment could greatly improve the treatment, protect myocardial function, and relieve inflammatory response in children with VMC.

## 1. Introduction

Viral myocarditis (VMC) is a kind of infectious myocardial disease in which viral infection triggers myocardial interstitial inflammatory cell infiltration and adjacent myocardial cell necrosis, further leading to cardiac dysfunction and other systemic damage [1]. It is pathologically characterized by necrosis and degeneration of cardiomyocytes and sometimes involves the pericardium or endocardium. Many common viruses, such as *Coxsackievirus*, *echovirus*, *poliovirus*, and *adenovirus*, can cause VMC [2]. VMC in children has an annual incidence ranging from 0.26 to 2 cases per 100,000 children [3], and 10 to 22 people suffer from VMC per 100,000 [2]. Clinically, patients commonly present with fatigue, limited mobility, palpitations, and chest pain, but the severity of symptoms varies among individuals. A few critically ill patients may develop heart failure and cardiogenic shock with a high mortality rate, and *Coxsackievirus B* infection is prevalent in the neonatal population [4].

The current main treatment of VMC includes antiviral, myocardial nutritional support, and immunomodulatory measures, but conventional treatment often fails to effectively control the disease, and thus, the recurrence rate is high [5]. Phosphocreatine, a supplement to adenosine triphosphate (ATP) deficiency, can increase energy-rich phosphate compounds in the myocardium to reduce ATP consumption and oxygen-free radical injury, thereby protecting myocardial tissues [6, 7]. Vitamin C, working as a vital free radical scavenger, can not only inhibit the release of superoxide free radicals from inflammatory cells but also alleviate the attack of oxygen free radicals on polyunsaturated fatty acids in lipids and damage to myocardial cells [8]. Vitamin C has definite efficacy and mild toxicity [9]. At present, many studies have reported the efficacy of creatine phosphate sodium (CPS) and/or vitamin C in the treatment of VMC in children, but there is still a lack of systematic reports.

This study aimed to conduct a systematic review to investigate the clinical utility of CPS and/or vitamin C in the treatment of VMC in children.

## 2. Materials and Methods

### 2.1. Literature Search Strategy

A literature search was performed on PubMed, Web of Science, Embase, China National Knowledge Infrastructure, and Wanfang databases, with a time span from January 2013 to January 2022. The keywords were “Viral myocarditis,” “creatine phosphate sodium,” and/or “vitamin C.” The corresponding Chinese translation of the search strategy was used for the Chinese database search.

### 2.2. Inclusion Criteria

The inclusion criteria are as follows: (1) study type (randomized controlled trials (RCTs) comparing the clinical efficacy of conventional treatment (CT) alone and CT combined with CPS and/or vitamin C for children with VMC); (2) study subjects (children confirmed with VMC according to their clinical manifestations, myocardial injury markers, etiological detection, and imaging examinations such as electrocardiogram and echocardiography); (3) intervention measures (control group having CT and observation group receiving CT combined with CPS and/or vitamin C); and (4) outcome measures, at least including one of the following (treatment effective rate, cardiac troponin-I (cTnI), creatine kinase isoenzyme (CK-MB), lactate dehydrogenase (LDH), aspartate aminotransferase (AST), tumor necrosis factor-*α* (TNF-*α*), and superoxide dismutase (SOD)).

### 2.3. Exclusion Criteria

Exclusion criteria are as follows: (1) studies with interventions that did not involve CPS and/or vitamin C and non-RCTs and studies without clear diagnostic criteria; (2) studies with vague and missing data, or with data that could not be converted and combined, or with key data that were not obtainable after communication with the authors of the literature; and (3) reviews, case reports, and conference papers.

### 2.4. Literature Screening and Data Extraction

Duplicate literature was first automatically eliminated by importing the articles into the EndNote software and then manually checked again. The remaining literature underwent independent secondary screening by two researchers in strict accordance with the established inclusion and exclusion criteria. The eligible articles were screened by reading the title, abstract, or full text, and the required relevant data was extracted. The required data included the following: title, first author, publication time, study design, sample size of the study subjects, interventions, and outcome of measures. In case of disagreement between two researchers, a third researcher was introduced to reach a consensus.

### 2.5. Statistical Analysis

In this study, the Stata 16.0 statistical software was used to analyze the relevant data of the included articles. Binary variables were expressed as odds ratio (OR), while continuous variables as standardized mean difference (SMD) with 95% confidence intervals (CI). The statistical heterogeneity among studies was evaluated using the chi-square test and *I*^2^ statistic. For *P* ≥ 0.05 and *I*^2^ ≤ 50%, which indicated no significant difference in heterogeneity, the fixed-effects model was adopted to combine effect sizes; otherwise (*P* < 0.05 or *I*^2^ > 50%), the random-effects model was selected. Sensitivity analysis was used to verify the reliability of the meta-analysis results, and funnel plots were constructed to assess publication bias analysis using the Begg method. Statistical differences were indicated by *P* < 0.05.

## 3. Results

### 3.1. Literature Search Results

In total, 723 articles were preliminarily searched. With 307 repeated and unqualified literature excluded, the titles and abstracts of the remaining studies were read to exclude 314 studies. Further 102 articles were submitted to screening by reading the original text, and 83 literature that did not meet the criteria were excluded according to the inclusion criteria. Finally, 19 studies were included in this present study [10–28]. The literature screening process and results are shown in Figure 1. A total of 1,957 VMC patients were included, with 968 patients in the control group and 989 patients in the observation group. The relevant basic characteristics of the literature are shown in Table 1.

### 3.2. Clinical Efficacy of Creatine Phosphate Sodium and/or Vitamin C for Viral Myocarditis in Children

#### 3.2.1. Meta-Analysis Results of Effective Rate after Treatment

A total of 11 studies [10–12, 16, 17, 19, 21, 24, 26–28] compared the treatment effective rate of the two groups of children with VMC. The fixed-effects model was used to combine the effect size because of no significant heterogeneity (*I*^2^ = 0.0% and *P* = 1.000). Meta-analysis results showed that the treatment effective rate in the observation group was significantly higher than in the control group (OR = 3.60, 95% CI (2.55, 5.07), *P* < 0.001, Figure 2(a)).

To ensure the reliability of the results, sensitivity analysis was carried out by eliminating each study one by one to find the source of heterogeneity, and still, the fixed-effects model was used for calculation. As shown in Figure 2(b), the newly obtained results were not significantly different from the original meta-analysis results, indicating that the meta-analysis results were robust and credible. Begg's funnel plot was used for publication bias analysis. The scatter points on both sides in the funnel plot were roughly distributed on the top and showed asymmetric distribution, indicating that there might be some publication bias in the included studies (Figure 2(c)).

#### 3.2.2. Meta-Analysis of Myocardial Injury Markers after Treatment

cTnI was compared between the two groups in 11 articles [11, 12, 14, 16–19, 23–26], CK-MB in 14 studies [10–12, 14, 16–26], LDH in 13 RCTs [10, 12, 14–17, 20–26], and AST in 8 articles [11, 15–17, 21, 22, 24, 26]. No significant heterogeneity was found among the studies (cTnI, *I*^2^ = 96.6%, *P* = 0.001; CK-MB, *I*^2^ = 96.6%, *P* = 0.001; LDH, *I*^2^ = 94.3%, *P* = 0.001; and AST, *I*^2^ = 97.7, *P* = 0.001), so the random-effects model analysis was used. In comparison with the controls receiving CT only, children with VMC treated with CT combined with CPS and/or vitamin C had lower levels of cTnI (SMD = −2.63, 95% CI (−3.51, −1.76), and *P* < 0.001), CK-MB (SMD = −2.78, 95% CI (−3.53, −2.03), and *P* < 0.001), LDH (SMD = −1.95, 95% CI (−2.49, −1.42), and *P* < 0.001), and AST (SMD = −0.87, 95% CI (−1.84, 0.09), and *P* = 0.076); there were statistically significant differences in these myocardial markers except AST (Figures 3(a)–3(d)).

For sensitivity analysis of cTnI, CK-MB, LDH, and AST after treatment in the two groups, the data were logarithmically transformed using the random-effects model, and individual studies were eliminated one by one. According to the newly combined results, heterogeneity of cTnI might be attributed to the studies by Qingyue Yu [12] and Chunli Li [16], for CK-MB to the study by Huimin Yang [19], LDH to the study by Quan Yuan [26], and AST to the studies by Jinghui Li [17] and Jun Liao [21] (Figures 4(a)–4(d)). Subsequently, the RCTs reporting cTnI, CK-MB, LDH, and AST were analyzed for publication bias. The scatter points on both sides of the funnel plot showed asymmetric distribution, indicating that the included studies had publication bias, which might be related to the small sample size of some studies or the low quality of the included literature (Figures 5(a)–5(d)).

#### 3.2.3. Meta-Analysis of Inflammatory Parameters after Treatment

A total of 5 articles [10, 21, 25, 27, 28] compared TNF-*α* in two groups of pediatric patients with VMC and 4 [13, 19, 20, 27] compared SOD with significant heterogeneity among studies (TNF-*α*, *I*^2^ = 87.4%, *P* = 0.001; SOD, *I*^2^ = 89.7%, *P* = 0.001). The results based on the random-effects model showed that TNF-*α* (SMD = −3.90, 95% CI (− 4.47, − 3.06), and *P* < 0.001; Figure 6(a)) in the observation group was significantly lower than in the control group and the former also had higher levels of SOD (SMD = 2.48, 95% CI (1.64, 3.33), and *P* < 0.001; Figure 6(b)).

Further, sensitivity analysis was performed for TNF-*α* and SOD after treatment in the two groups. The findings after removing each study one by one revealed that the study by Suyuan Hu [27] could be the source of heterogeneity of TNF-*α*, while that of Yuantao Lin [13] could be the source of heterogeneity of SOD (Figures 7(a)–7(b)). Subsequently, publication bias analysis was performed for TNF-*α* and SOD after treatment in patients, respectively. The scatter points were mainly distributed at the bottom of the funnel plot and in asymmetric distribution, indicating that there may be some publication bias. The reason for bias could be because the sample size of some studies was too small (Figures 8(a)–8(b)).

## 4. Discussion

In the second half of the twentieth century, Fiedler pointed out that the main histopathological characteristic of myocarditis was the presence of intramyocardial inflammatory infiltrates [29]. Bell et al. [30] and the 1987 consensus [31] reinforced this concept and defined myocarditis as a disease characterized by inflammatory cell infiltrates in the heart. In 1956, Javett et al. first confirmed that *Coxsackievirus B3* caused an epidemic of myocarditis in 10 infants at a maternity home in Johannesburg, South Africa [32]. Since then, there have been increasing researchers isolating viruses from the myocardium of dead patients, and promising advances were made in the pathogenesis, diagnosis, and treatment of VMC due to the establishment of mouse models of VMC, development of laboratory diagnostic techniques, and progress in molecular biology, biochemistry, immunology, and other disciplines [33–36]. Although the pathogenesis of this disease is not fully understood, VMC was confirmed to be directly affected by viruses, host genetic background, immune response, and oxidation [37]. Reactive oxygen-induced lipid peroxidation plays an important role in the damage of myocardial cells among the four aspects.

The blocking effect of high-dose vitamin C and the myocardial protective effect of CPS have been confirmed in many reports [8, 11, 18]. In this present study, we systematically assessed the clinical efficacy of CPS and/or vitamin C in treating VMC in children. By searching the relevant databases in Chinese and English, a total of 19 studies were included for meta-analysis, avoiding the disadvantages of small sample sizes and low statistical power of single studies. Compared with the control group who underwent CT therapy, we found the observation group receiving CPS and/or vitamin C had better performance in effective rate and myocardial markers (cTnI, CK-MB, LDH, and AST) in children with VMC. This is consistent with the research results of other researchers. Wu Shihua et al. included 17 literature for meta-analysis and reported that CPS combined with vitamin C for VMC was superior to CT in overall effective rate, serum creatine kinase, LDH, and cTnI [38]. Serum CTnI concentration in the pediatric viral VMC group has been proved to be higher than that in the controls in a meta-analysis on the diagnostic value of cTnI for VMC [39]. CK-MB and serum LDH also have important significance in the early diagnosis of myocardial injury. Although the sensitivity of cTnI is not high, it has demonstrated a high specificity in diagnosing VMC. In addition, we compared and analyzed the inflammatory parameters after CPS and/or vitamin C treatment for VMC in children; compared with the control group, TNF-*α* after treatment was lower, and SOD was higher in the observation group. A meta-analysis by Chen et al. found that intravenous vitamin C for VMC in children was also superior to the control group in TNF-*α* levels and CK-MB and LDH levels [40]. In 1993, Cui Xiaodai reported that 150 to 200 mg/kg of intravenous vitamin C could give full play to its antioxidant effect and this concentration of vitamin C would not destroy myocardial cells [41]. The antioxidant effect of vitamin C reduces oxygen free radicals and protects myocardial cells.

However, there are some limitations to this study. Since there is little English literature on CPS and/or vitamin C in the treatment of VMC, most of the included literature in this study was in Chinese and might have led to a certain level of publication bias. Second, some differences in the intervention measures of the control and observation groups were observed in the included literature and the severity of VMC in patients in different studies. Such differences can have a certain impact on the reliability of the results of this meta-analysis. Thus, multicenter studies with larger sample sizes, and high quality are still needed to further confirm these findings.

## 5. Conclusion

In summary, compared with CT alone, CT combined with CPS and/or vitamin C could improve the effective rate of VMC treatment in children. These findings may help to guide and standardize the treatment of this disease. However, high-quality RCTs with larger sample size performed at multiple centers and with rigorous design should be performed in the future to provide more accurate and reliable clinical evidence for this conclusion.

## Figures and Tables

**Figure 1:** Flow chart of literature screening.

**Figure 2:** Meta-analysis results of treatment effective rate in children with viral myocarditis in the two groups. (a)–(c) Forest plot (a), sensitivity analysis (b), and funnel plot (c) of the treatment effective rate.

**Figure 3:** Forest plots to compare myocardial markers in children with viral myocarditis in the two groups. (a) Cardiac troponin-I (cTnI); (b) creatine kinase isoenzyme (CK-MB); (c) lactate dehydrogenase (LDH); and (d) aspartate aminotransferase (AST).

**Figure 4:** Sensitivity analysis of myocardial markers in children with viral myocarditis in the two groups. (a) Cardiac troponin-I (cTnI); (b) creatine kinase isoenzyme (CK-MB); (c) lactate dehydrogenase (LDH); and (d) aspartate aminotransferase (AST).

**Figure 5:** Funnel plots of myocardial markers in children with viral myocarditis in the two groups. (a) Cardiac troponin-I (cTnI); (b) creatine kinase isoenzyme (CK-MB); (c) lactate dehydrogenase (LDH); and (d) aspartate aminotransferase (AST).

**Figure 6:** Forest plots of inflammatory markers in children with viral myocarditis in the two groups. (a) Tumor necrosis factor-*α* (TNF-*α*) and (b) superoxide dismutase (SOD).

**Figure 7:** Sensitivity analysis of inflammatory markers in children with viral myocarditis in the two groups. (a) Tumor necrosis factor-*α* (TNF-*α*) and (b) superoxide dismutase (SOD).

**Figure 8:** Funnel plots of inflammatory markers in children with viral myocarditis in the two groups. (a) Tumor necrosis factor-*α* (TNF-*α*) and (b) superoxide dismutase (SOD).

**Table 1:** Basic characteristics of included literature.

Study	Year	Intervention	No. participants (Ob/Co)	Age(years)		Gender (male/female)		Study design	Outcome measured
				Observation group	Control group	Observation group	Control group		
Baoqin Tao [10]	2021	Vitamin C combined with immunoglobulin	63/45	7.35 ± 0.36	7.24 ± 0.57	33/30	24/21	RCT	①③④⑥
Xiaojie Yang [11]	2021	Vitamin C combined with sodium creatine phosphate	40/40	6.32 ± 1.68	6.19 ± 1.83	21/19	21/19	RCT	①②③⑤
Qingyue Yu [12]	2020	Vitamin C combined Creatine phosphate sodium	31/31	6.42 ± 1.31	6.35 ± 1.22	20/11	21/10	RCT	①②③④
Yuantao Lin [13]	2015	Phosphate sodium and captopril	40/40	4.6 ± 2.5	4.5 ± 2.8	21/19	20/20	RCT	①⑦
Junying Sun [14]	2015	Creatine phosphate sodium and thymopeptides	37/37	6.05 ± 1.56	6.85 ± 1.23	—	—	RCT	①②③
Yuan Liu [15]	2021	Creatine phosphate sodium and immunoglobulin	67/67	4.79 ± 1.40	4.58 ± 1.66	34/33	36/31	RCT	④⑤
Chunli Li [16]	2019	Ulinastatin combined with creatine phosphate sodium	80/75	8.63 ± 3.76	8.54 ± 3.15	60/20	56/19	RCT	①②③④⑤
Jinghui Li [17]	2021	Gamma globulin combined with creatine phosphate	62/59	7.58 ± 2.16	7.64 ± 2.23	35/27	34/25	RCT	①②③④⑤
Ruibo Gao [18]	2018	Vitamin C combined immunoglobulin	38/38	3-11	3-12	22/16	23/15	RCT	②③
Huimin Yang [19]	2021	Sodium fructose diphosphate combined with creatine phosphate acupuncture	42/42	8.21 ± 2.13	8.49 ± 2.26	24/18	25/17	RCT	①②③⑦
Yizhen Gong [20]	2017	Adenosine cyclophosphate combined with vitamin C	44/44	7-12	6-12	25/19	24/20	RCT	③④⑦
Jun Liao [21]	2016	Adenosine cyclophosphate combined with vitamin C	55/55	7.28 ± 0.82	7.41 ± 0.86	33/22	32/23	RCT	①③④⑤⑥
Xiu Chang [22]	2016	Adenosine cyclophosphate combined with vitamin C	48/48	7.5 ± 2.6	7.2 ± 2.3	27/21	26/22	RCT	④⑤
Caihong Li [23]	2016	Astragalus granules combined with vitamin C	68/73	6.29 ± 2.17	6.75 ± 2.45	36/32	40/33	RCT	②③④
Yujia Li [24]	2018	Creatine phosphate sodium combined with ribavirin	48/48	6.95 ± 1.32	6.91 ± 1.27	28/20	25/23	RCT	①②③④⑤
Yue Jiang [25]	2020	Sodium creatine phosphate combined with vitamin C	36/36	7.16 ± 1.92	6.95 ± 1.89	15/21	16/20	RCT	②③④⑥
Quan Yuan [26]	2016	Sodium creatine phosphate combined with Xinjikang granules	80/80	9.26 ± 1.24	9.32 ± 1.37	46/34	44/36	RCT	①②③④⑤
Suyuan Hu [27]	2015	Vitamin C combined with adenosine cyclophosphate	65/65	—	—	34/31	33/32	RCT	①⑥⑦
Meng Wang [28]	2020	Vitamin C combined with immunoglobulin	45/45	8.30 ± 0.97	8.39 ± 0.91	24/21	23/22	RCT	①⑥

Note: ob: observation group; co: control group; RCT: randomized controlled trial; ①: treatment effective rate, ②: cardiac troponin-I, ③: creatine kinase isoenzyme, ④: lactate dehydrogenase, ⑤: aspartate aminotransferase, ⑥: tumor necrosis factor-*α*, ⑦: superoxide dismutase.

## Data Availability

The data that support the findings of this study are available from the authors upon reasonable request.

## Abbreviations

CPS: Creatine phosphate sodium
VMC: Viral myocarditis
RCTs: Randomized controlled trials
ATP: Adenosine triphosphate
CT: Conventional treatment
cTnI: Cardiac troponin-I
CK-MB: Creatine kinase isoenzyme
LDH: Lactate dehydrogenase
AST: Aspartate aminotransferase
TNF-*α*: Tumor necrosis factor-*α*
SOD: Superoxide dismutase
OR: Odds ratio
CI: Confidence intervals.

## Additional Points

*Author details.* Department of Pediatrics, General Hospital of Northern Theater Command. No.5 Guangrong Street, Heping District, Shenyang 110812, China.

## References

[1] Richardson P. (1995). Report of the 1995 World Health Organization/International Society and Federation of Cardiology Task Force on the definition and classification of cardiomyopathies. *Circulation*.

[2] Olejniczak M., Schwartz M., Webber E., Shaffer A., Perry T. E. (2020). Viral myocarditis-incidence, diagnosis and management. *Journal of Cardiothoracic and Vascular Anesthesia*.

[3] Matsuura H., Ichida F., Saji T. (2016). Clinical features of acute and fulminant myocarditis in children-2nd Nationwide Survey by Japanese Society of Pediatric Cardiology and Cardiac Surgery. *Circulation Journal*.

[4] Wu R. Z. (2012). Research progress in pathogenesis of viral myocarditis in children. *Chinese Journal of Practical Pediatrics*.

[5] Ye T., Yue Y., Fan X., Dong C., Xu W., Xiong S. (2014). M cell-targeting strategy facilitates mucosal immune response and enhances protection against CVB3-induced viral myocarditis elicited by chitosan-DNA vaccine. *Vaccine*.

[6] Wang Z. Q. (2013). The effect observation of creatine phosphate in the treatment with viral myocarditis of children 70 cases. *Chongqing Medicine*.

[7] Su Cao, Hui-hui Yao, Feng Niu (2013). Effect of creatine phosphate sodium in treatment of viral myocarditis in infants. *Journal of Xinxiang Medical University*.

[8] Guo H. J. H. R., Xiong Y. J. (2013). Effect of high dose vitamin C on herpes simplex keratitis. *Chongqing Medicine*.

[9] Pan X. B., Sun J. H., Gao Q. (2012). Progress in diagnosis and treatment of viral myocarditis in children. *Chinese Journal of Laboratory Diagnosis*.

[10] Tao B. Q., Wang J. Q., Yang H. M. (2015). Effect of vitamin C combined with immunoglobulin on myocardial injury and myo-cardial remodeling in children with viral myocarditis. *Northwest Pharmaceutical Journal*.

[11] Yang X. J. (2014). Effects of high-dose vitamin C combined with sodium creatine phosphate on serum BNP,cTnI and CK-MB levels in children with viral myocarditis. *Heilongjiang Medicine And Pharmacy*.

[12] Yu Q. L. (2016). Effect of vitamin C combined with creatine phosphate sodium on clinical efficacy and myocardial enzyme levels in children with viral myocarditis. *Xinxueguanbing Fangzhi Zhishi*.

[13] Lin Y. T., Zeng X. L., Chen L., Xu Y., Zhang Y. (2015). Effect of phosphate sodium and captopril in the treatment of children with viral myocarditis. *Chinese Journal of Primary Medicine and Pharmacy*.

[14] Sun J. Y. (2014). Effect of thymosin combined with creatine phosphate sodium on viral myocarditis in children. *Medicine and Health Care*.

[15] Liu Y. (2015). Effect of creatine phosphate combined with immunoglobulin on myocardial enzymes in children with viral myocarditis. *Capital Medicine*.

[16] Li C. L., Jia L. B., Gao J., Wang Z. Z., An X. J. (2019). The efficacy observation of ulinastatin combined with creatine phosphate sodium in pediatric viral myocarditis. *European Review for Medical and Pharmacological Sciences*.

[17] Li J. H., Li T. T., Wu X. S., Zeng D. L. (2021). Effect of gamma globulin combined with creatine phosphate on viral myocarditis. *American Journal of Translational Research*.

[18] Gao R. B., Jiang H. (2018). Clinical value of high-dose VitC + immunoglobulin for the treatment of viral myocarditis in children. *Journal of Hainan Medical University*.

[19] Yang H. M. (2017). Observation of the effect of sodium fructose diphosphate combined with creatine phosphate acupuncture on viral myocarditis in children. *Harbin Medical Journal*.

[20] Gong Y. Z., Li S. C. (2017). Study on the protective effect of adenosine cyclophosphate combined with vitamin C antiviral therapy on myocardial injury in children with viral myocarditis. *Journal of Hainan Medical University*.

[21] Liao J. (2015). Effect of adenosine cyclophosphate combined with vitamin C therapy on electrocardiogram and serum indexes of children with viral myocarditis. *Journal of Hainan Medical University*.

[22] Chang X., Jiu L. H. (2016). Adenosine cyclophosphate combined with vitamin C treatment of children with viral myocarditis and the effect on cellular immunefunction. *Journal of Hainan Medical University*.

[23] Li C. H. (2016). Protective effect of creatine phosphate sodium, vitamin C combined with antiviral therapy on myocardial damage in children with viral myocarditis. *Journal of Hainan Medical University*.

[24] Li Y. J., Lu W., Du K. (2018). Clinical efficacy of creatine phosphate sodium combined with ribavirin in treating infantile viral myocarditis and its effect on myocardial enzyme levels in children. *Journal of Jilin University(Medicine Edition)*.

[25] Jiang Y., Wang Q. (2017). Efficacy of sodium creatine phosphate combined with vitamin C in the treatment of viral myocarditis in children. *Chinese Journal of Hemorheology*.

[26] Yuan Q., Zhang P. (2016). Analysis on effectiveness of Xinjikang granules combined with creatine phosphate sodium for treating children with viral myocarditis. *Chongqing Medicine*.

[27] Hu S. Y. (2018). The application of vitamin C combined with adenosine cyclophosphate in children with viral myocarditis. *Journal of Bengbu Medical College*.

[28] Wang M., Zhang X., Xing S. H., Ma Y. (2016). Effects of vitamin C combined with immunoglobulin on myocardial injury and miR-21,miR-451 in children with viral myocarditis. *Journal of Clinical and Experimental Medicine*.

[29] Sanders V. (2016). Viral myocarditis. *The American Journal of Pathology*.

[30] Bell R. W., Murphy W. M. (1967). Myocarditis in young military personnel. Herpes simplex, trichinosis, meningococcemia, carbon tetrachloride, and idiopathic fibrous and giant cell types. *American Heart Journal*.

[31] Aretz T. H. (1986). Myocarditis. A histopathologic definition and classification. *The American Journal of Pathology*.

[32] SN J., WJ P. (1956). Myocarditis in the new newborn infant; a study of an outbreak associated with Coxsackie group B virus infection in a maternity home in Johannesburg. *The Journal of Pediatrics*.

[33] Sainani G. S., Krompotic E., Slodki S. J. (1968). Adult heart disease due to the Coxsackie virus B infection. *Medicine*.

[34] Smith W. G. (1970). Coxsackie B myopericarditis in adults. *American Heart Journal*.

[35] Levi G. F., Proto C., Quadri A., Ratti S. (1977). Coxsackie virus heart disease and cardiomyopathy. *American Heart Journal*.

[36] Li Y., Bourlet T., Andreoletti L. Enteroviral capsid protein VP1 is present in myocardial tissues from some patients with myocarditis or dilated cardiomyopathy. *Circulation*.

[37] Sun J. H., Zhai S. B. (2017). Progress in the research on viral myocarditispathogenesis. *Journal of Clinical Pediatrics*.

[38] Wu S. H., Chen X., Wen J. X., Wu J. D. (2015). Systematic review of sodium creatine phosphate combined with vitamin C in the treatment of pediatric viral myocarditis. *Evaluation and Analysis of Drug-Use in Hospitals of China*.

[39] Hou Q. S. (2015). Meta-analysis on diagnostic value of cardiac troponin I for viral myocarditis in children. *Chinese Journal of General Practice*.

[40] Chen S., Zhao W., Zhang B. (2019). Clinical effect of intravenous vitamin C on viral myocarditis in children: a systematic review and meta-analysis. *Evidence-based Complementary and Alternative Medicine*.

[41] Ma P. R., Zhang Y. (2015). Progress and prospect of diagnosis and treatment of viral myocarditis in children. *Chinese Journal of Practical Pediatrics*.

